The article "Early Detection of Forest Fire Using Mixed Learning Techniques and UAV" was published in 2022. Journal: Comput Intell Neurosci.

# Early Detection of Forest Fire Using Mixed Learning Techniques and UAV

**DOI:** 10.1155/2022/3170244

**Published:** 2022-07-09

**Authors:** Varanasi LVSKB Kasyap, D. Sumathi, Kumarraju Alluri, Pradeep Reddy CH, Navod Thilakarathne, R. Mahammad Shafi

**Affiliations:** ^1^VIT-AP University, Amaravati, Andhra Pradesh 522237, India; ^2^Faculty of Technology, University of Colombo, Colombo, Sri Lanka; ^3^College of Engineering and Technology, Tepi Campus, Mizan-Tepi University, Mizan Teferi, Ethiopia

## Abstract

Over the last few decades, forest fires are increased due to deforestation and global warming. Many trees and animals in the forest are affected by forest fires. Technology can be efficiently utilized to solve this problem. Forest fire detection is inevitable for forest fire management. The purpose of this work is to propose deep learning techniques to predict forest fires, which would be cost-effective. The mixed learning technique is composed of YOLOv4 tiny and LiDAR techniques. Unmanned aerial vehicles (UAVs) are promising options to patrol the forest by making them fly over the region. The proposed model deployed on an onboard UAV has achieved 1.24 seconds of classification time with an accuracy of 91% and an F1 score of 0.91. The onboard CPU is able to make a 3D model of the forest fire region and can transmit the data in real time to the ground station. The proposed model is trained on both dense and rainforests in detecting and predicting the chances of fire. The proposed model outperforms the traditional methods such as Bayesian classifiers, random forest, and support vector machines.

## 1. Introduction

Recent advancements in technology have overwhelmingly shaped society, the economy, and the environment. With the help of the various state-of-art technologies such as IoT, blockchain, AI, geospatial mapping, and so on, leading to the fifth industrial revolution, which focuses more on solving climate goals in line with the revolution [1]. New requirements in the ecological environment arise due to the expeditious development of society. Among the various natural disasters, fire hazard seems to own the characteristics of spreading, and also, it becomes very challenging to control, and thus, it results in heavy destruction that might be irrevocable [2–4]. Over the past few years, there is a tremendous increase in the count, occurrence, and severity of wildfires across the world that has created a great impact on the economy and ecosystem of the country. There are various techniques such as watchtowers, spotter planes, infrared, aerial patrols, and automatic detection systems to detect fire events [1]. There is no need for the exposure of humans to perilous activities when remote sensing is deployed [5]. Various techniques are as follows:

- Usage of the satellite images to observe, detect, and report fire events
- Implementation of the wireless sensor networks to observe the fire events exist in all areas.

The article "Early Detection of Forest Fire Using Mixed Learning Techniques and UAV" was published in 2022. Journal: Comput Intell Neurosci.

Yet there are certain limitations associated with the satellite images [6–8]. It has an inadequate resolution, and hence, the data pertinent to the corresponding area would be taken as an average, and it is restricted to a particular pixel that results in the detection of small fires. The predominant limitation is that the satellites cover only a limited area and require a preprocessing time before the resurvey of the same region. The other limitations such as the shortage of real-time data and inadequate precision are inapt for persistent monitoring. There is a need for the infrastructure in advance if WSNs are deployed [4]. There is more chance for the destruction of the sensors during the fire, and this might lead to more expensive restoration of the sensors [9]. Several factors such as the static nature of the sensors, their coverage, difficulty in maintenance, the deficit in power independence, and nonscalability are the reasons for the sensor networks to limit their efficiency. Therefore, unmanned aerial vehicles (UAVs) are proposed to overcome the limitations. The sovereignty, less cost, autonomous, and flexibility make the UAV technology the best choice for fire management efforts in the wildland. There are researchers who put more effort into focusing on the development of frameworks and techniques that could be associated with UAVs. The motive of the implementation of UAV is to detect the fire and its coverage in an optimal manner [3, 10]. The aim of this work is to develop a model to detect the fire and its coverage area, and in addition, it also observes the fire in the low region.  Section 2 describes the related works associated with fire detection.  Section 3 elaborates on the proposed model and architecture. Finally, the results and discussion to prove the proposed model are covered in Section 4. The last section concludes with a summary and future scope.

## 2. Related Works

Detection of forest fire and smoke in wildland areas is done through remote sensing-based methods such as satellites, high-resolution static cameras fixed on the ground, and unmanned aerial vehicles (UAVs).

The limitations of the satellites [11] are described as follows:

- Images that are captured through the satellites have poor resolution, and hence, it becomes difficult to detect the particular area
- Continuous information about the status of the forest could not be obtained due to the restrictions in the monitoring of forests
- Weather might not be stable in all situations as it might vary, and thus, it results in the collection of noisy images

Optical/thermal cameras deployed on the observation towers together with the other sensors such as smoke, temperature, and humidity sensors might detect the hazards in the closed environment rather than in the open environment as these sensors need vicinity to the fire or smoke. The information obtained through these sensors is not appropriate. Distance covered by these methods could be limited, and to cover a large area, more sensors have to be deployed that might incur expenses. Through the deployment of UAV, large areas could be covered, and the images with high spatial and temporal resolutions could be captured properly. The operational cost is very low when compared with the other methods.

The article "Early Detection of Forest Fire Using Mixed Learning Techniques and UAV" was published in 2022. Journal: Comput Intell Neurosci.

In [12], detection of forest fire is done through the deployment of YOLOv4 to UAV-based aerial images. The initial phase of the process is that the authors developed the hardware platform and proposed the YOLOv4 algorithm. Frame detection rate through this method obtained is 3.2 fps, and the recognition rate achieved is 83%. This works when the intensity of the fire is huge. The limitation of this algorithm is that the detection rate is very less in the small fire-spot areas. The authors have made use of the NetImage classifier that has the combination of Yolov5 and EfficientDet. The data set used comprises 10,581 images of which 2,976 images are categorized as forest fire and 7,605 as nonfire images. The model undergoes an adequate training process, and an accuracy of 99.6% has been obtained with the 476 fire images, and for 676 images that looked similar to images that display fire, the accuracy achieved was 99.7%. Yet the limitation is that it does not detect the smoke since it is needed in the initial stage of the detection process.

In this work [2, 13], the detection of forest fire is done automatically with the help the image processing methods. The principle behind the proposed work is that the image brightness and motion clues are used with the image processing techniques that depend on histogram-based segmentation. Initially, the hot objects are identified, and they are recognized as the candidate regions. Next, the motion vectors of the candidate regions are computed based on the optical flow. Furthermore, the vectors are used to isolate the fires from the other systems that might look similar to the fire. Tracking of fire from IR images is done through the Blob counter technique and morphological operations. Results have shown that the proposed method does the extraction and detection of the fire pixels effectively. Extraction of the background from the video and determination of the proper motion regions by analyzing the difference between the subsequent frames is done through the ViBe method. Several functions such as median filtering, color space conversion, Otsu threshold segmentation, morphological operations, and Blob counter are used [3, 14]. The fire and smoke areas are identified through the extraction of both static and dynamic features. Caffemodel that works based on deep learning is the principle that is used to detect fire and smoke areas. Apart from these, the degree of irregularity of the smoke and fire is also analyzed.

The article "Early Detection of Forest Fire Using Mixed Learning Techniques and UAV" was published in 2022. Journal: Comput Intell Neurosci.

The false alarm rate is reduced, and the original position of the fire is also identified in this work by considering that each and every frame image of the video is partitioned into 16 × 16 grids and the occurrences of each part of the fire and smoke are recorded. The evidence is collected so as to decide on the final detection. From the experimental results, it is shown that the loss has been reduced, and fire and smoke are detected. Various researchers have worked in exploring forest fire detection in a diversified manner. In [4, 15–17], fuzzy logic-based smoke detection and segmentation schemes are introduced along with the principle of the extended version of the Kalman filter. Segmentation of smoke is done with fuzzy logic, and thus, the prospects of occurrence of smoke are identified. This is done by observing the difference in the background images and the intensity. The extended version of the Kalman filter is used to eradicate the effects that might be due to the disparities in the environmental conditions by reshaping the inputs of the fuzzy smoke detection rule. The authors [18] have worked on the technique that works based on the principle of color and motion. In this work, the UAV is equipped with obscure and an optical camera which is used to detect the forest fire.

Cameras mounted are used to procure free flame infrared and visual pictures. Images could be combined with the landscape information and meteorological data to observe the forest fire. With this technique, the false alert rates of forest fire detection are decreased. A novel method based on the new color index named Forest Fire Detection Index (FFDI) has been proposed in [1, 19–21]. Index computation is done based on vegetation categorization. The tones of the flame and smoke are also detected that in addition is used to form the regions of interest (RoI). The precision of the detection is found to be 96.82% for the image sizes of 960 × 540 pixels that have been processed in 0.447 seconds. The frame considered during the experimental investigations was 22 frames/second for smaller images, and it has been extended to 54 frames/second. The precision rate at the early detection stage has been observed as 96.62%. A deep learning framework named Fire-Net has been devised in [9]. Here, the model is trained on Landsat-8 imagery so that the detection of the active fires and burning biomass is done. The images that are obtained have been represented effectively with the help of optical fusion and thermal modalities. Extraction of a deep set of features is facilitated by providing more attention to the residual convolution and discrete convolution blocks. From the experiments, the overall accuracy is 97.35%, and the model is robust in the detection of small fires. Continuous monitoring of the potential areas that might be prone to fire should be monitored. In this work [22–25], the design of UAVs has been done based on the advantages of AI. Furthermore, the onboard processing abilities have also been equipped. The inputs to the model are the still images or the video input that are captured through the cameras mounted on the drone [14, 26, 27]. The drones are supported by both fixed and the rotary-wing. The fixed-wing drone is used to monitor the area frequently. It covers an altitude from 350 m to 5,500 m, and there might be a chance of reporting a false alarm. As soon as the fixed-wing drone detects the fire, an alarm is triggered that in turn stimulates the rotary-wing drone. With the help of GPS coordinates, it then examines the area. The second drone decides whether to trigger the alarm based on its observations. The main advantage of the second drone is to decrease the false alarm rate. Many research works have been carried out for detecting fire through IR images, whereas a few works are done on UAV platforms [28, 29].

The article "Early Detection of Forest Fire Using Mixed Learning Techniques and UAV" was published in 2022. Journal: Comput Intell Neurosci.

From the various inferences, it has been understood that most of the researchers have worked to increase the accuracy, and the area coverage was until 1,500 meters to the maximum. To provide more accuracy and precision, the 3D modeling of data is required, and further visualization of forest fire images could be made very easy for interpretation. The objective of this work is to deploy an efficient and robust detection fire in the early stage. Hence, a deep learning model is required so that the boundary region could be extended, and the 3D modeling images must be considered for the prediction process to augment the accuracy. The contributions in this work are as follows:

- An efficient and robust 3D modeling is used to augment the accuracy of the detection.
- A deep learning technique YOLOv4 is combined with the Otsu method along with LiDAR. The key objective of utilizing the Otsu method is to repeat all the values of the threshold and evaluate the extent of the background and foreground pixels. The objective is to determine the threshold by examining the region of the spread, and it should be minimum.
- Traditional methodologies are found to be difficult for performing the sampling since the constraints are bound to the relative position. Hence, the orientation of the images is required, and that is obtained by computing the distance between the tree and other entities with the help of LiDAR.  Section 3 describes the proposed methodology.

## 3. Proposed Methodology

The flow of the proposed architecture is shown in Figure 1. The video input is captured from the camera, and the other inputs such as wind speed, wind directions, and IR image sensing are calculated using the sensors mounted on the UAV for navigation. These images are provided as input to the deep learning models, and it checks for the existence of the fire. The region is predicted clearly since there is a possibility of more projections of the images provided to the model due to the 3D modeling. Further detection is made, and the details are stored in the database for further.

### 3.1. Autonomous Drone Routing

#### 3.1.1. Drone Moment to the Target

In this whole operation, navigation of UAVs is significant to patrol the risk-prone areas and fire-detected areas. This work monitors the forest area with the help of the navigational analysis technique [27, 30]. To facilitate this, the drone makes the navigation. UAVs have the following three navigational features [31]:

- Awareness: This provides details about UAV's neighborhood obstacles. The data is collected using internal sensors
- Basic Navigation: Collisions are avoided, and the obstacles such as birds, trees, poles, and so on in the forest farms are detected
- Expanded Navigation: Advanced features such as pathway planning and depth deployment are included and play a crucial role in autonomous navigation

This categorization of features is shown in Figure 2 that could provide a better understanding of the navigation of UAVs.

On detection of fire with YOLOv4 tiny, the autonomous patrol in the affected area is found to influence the decisions that must be considered for stopping the fire. The visual servoing algorithm [8] operates for the autonomous drift of UAV towards the fire; it works as follows:

**Step 1 .**

The location of the fire is requested, and it is captured through the (YOLOv4 tiny-bounding box of fire). If the fire is detected, go for step 2.

**Step 2 .**

Calculate the step size depending on the location of the bounding box of fire that is relative to the midpoint of the frame, along with the direction.

The article "Early Detection of Forest Fire Using Mixed Learning Techniques and UAV" was published in 2022. Journal: Comput Intell Neurosci.

**Step 3 .**

Normalize the drone for drift by changing the roll and angle of pitch of the current state.

**Step 4 .**

Set the next set point to control the flight and iterate the process.

When the forest is very thick and it is in the GPS-denied area, UAV makes use of hybrid-localization methods to achieve the maximum performance of the task. Many research works [31, 32] suggest the simultaneous localization and mapping (SLAM) algorithm to use in GPS-denied areas. The solitary idea of SLAM is to process mapping and localization concurrently and recursively. Using the Kalman filter, SLAM overcomes the problem of feature evaluation. SLAM algorithms develop the landmark-based navigation system with the capability of virtual-map navigation; this became a typical technique for the drone-based navigation application.  Figure 3 given below depicts the structure of the proposed localization solution based on vision. This structure operates the space and features on two different levels. It has three main modules: (1) hybrid feature extraction, (2) generating map, and (3) hybrid localization. The feature extraction component combines two different methods to find a location at two scales. The map generation component performs feature compression and feature evaluation. The filters extract the most appropriate features using an info-theoretic method, then compress the features, and evaluate them.

#### 3.1.2. Technical Information of UAV

Flight planning is considered a salient feature in designing the architecture of UAVs [33]. This planning illustrates the division of mass on UAVs and provides a better understanding of the performance analysis of UAVs. Specifically, maximum take-off weights (MTOW) assess the UAV payload capacity at different heights above the ground. The payload of the UAV and the mass of onboard equipment are given in Table 1, and the components of the UAV are depicted in Figure 3. The battery used on the UAV reserves the UAV in GPS-enabled environments for 107 minutes of duration, whereas on the GPS-disabled environment, maximum flight time is 87 minutes.

Figure 4 displays the digital anemometer, manifold CPU, IR sensors, and 12K camera.

The total payload of the UAV is 6,825 grams. The thrust of the UAV is capable to fly with a 7,000-gram payload and is calculated as follows:

(1) $$\begin{array}{c} \tau \left(T\right)=\frac{\pi }{4}d^{2}\rho v\Delta v, \end{array}$$

where *τ* = thrust of UAV, *d* = distance of propeller = 0.6556 m, *ρ*= air density (1.225 m kg/cubic meter), and *v* = aerial velocity at propeller (m/s) = 1/2∆v.

The power of the UAV is as follows:

(2) $$\begin{array}{c} P\left(W\right)=\frac{\tau \left(\Delta v\right)}{2},\\ Ρ\left(W\right)=\text{PropellerConstant}*{\left(\frac{rpm}{1000}\right)}^{\text{powerfactor}},\\ Ρ\left(W\right)=\mathrm{PropellerConstant*}d^{4}*p*rpm^{3}, \end{array}$$

where Propeller Constant = 1.11(for APC propeller) and *P* = pitch of propeller in air.

The article "Early Detection of Forest Fire Using Mixed Learning Techniques and UAV" was published in 2022. Journal: Comput Intell Neurosci.

The total mass lifted by the UAV is as follows:

(3) $$\begin{array}{c} m=\frac{\tau }{g},\\ m=\frac{{\left(\pi /2d^{2}\rho v\text{P}\right)}^{1/3}}{g}, \end{array}$$

where *g* = acceleration due to gravity.

Therefore, the maximum payload of the UAV is 8,000 grams.

Due to this high Power of UAV, it can take steep turns with a very low pitch angle in any direction and is capable to fly 350–400 m above the ground with a range of 3,000–4,000 m.

The time of flight of a UAV is calculated as follows:

(4) $$\begin{array}{c} T_{f}=c_{b}*\left(\frac{d_{b}}{AAD}\right), \end{array}$$

where *T*_*f*_ = time of flight in hours, *c*_*b*_ = capacity of battery (mAh), *d*_*b*_ = battery discharge, and *AAAD* = average ampere draw (ampere) of the UAV = AUW ^*∗*^ p/v.

### 3.2. Fire Detection and Fire Region Prediction

#### 3.2.1. Fire Detection in the Forest Region

A classic UAV can autonomously fly over the forest area and detect the forest fire and yaw around the burning forest fire area. The UAV is well equipped with IR sensors, a 12K camera for image accretion, and the onboard CPU, which can broadcast the real-time video of the forest fire to the ground station using the signals that are used for remote navigation. The ground station would diagnose and take necessary measures to stop the forest fire. In parallel, the ground station can also control the UAV by sending the operational commands.

The onboard CPU has good computation power to perform the forest fire detection using YOLOv4 tiny, which has good detection speed with well-grounded accuracy [11]. The YOLOv4 tiny model is divided into two layers, that is, the feature extraction layer and the processing layer. The feature extraction layer is the combination of the DarkNet and ResNet, similar to the feature-like pyramid network that has the convolutional layer, batch-normalization layer, and leaky ReLU layer. The problem of overfitting is shut out using batch normalization. The combination of the convolutional layer, batch-normalization layer, and leaky ReLU layer is called CBL. The combination of the convolutional layer, batch-normalization layer, and mish activation function is called CBM. The structure of CBL and CBM is shown in Figure 5.

The five max-pooling layers of the network of 2 ∗ 2 size with stride = 2 give the reduced feature map of 1/32th size of the original image. Since there is no fixed shape for fire and smoke, size is varied. YOLO layers are operated for the detection of fire using logistic regression. YOLOv4 tiny has an advantage of high speed and accuracy, due to its speed-up algorithm. The bounding boxes of YOLOv4 tiny can be achieved using region proposal network (RPN) [11]. Intersection over union (IOU) score is considered the metric and is used to obtain the bounding box. The distance measure for the clustering is given in

(5) $$\begin{array}{c} D\left(\text{boundingbox,centre}\right)=1-IOU\left(\text{boundingbox,centre}\right). \end{array}$$

The algorithm finds the bounding box as follows: image is captured by the camera, and the target is drawn to fix the center. The coordinate calculation of the image is given in Equation 2.

(6) $$\begin{array}{c} \left\{\begin{array}{c} BB_{x}=\sigma \left(p_{x}\right)+c_{x}\\ BB_{y}=\sigma \left(p_{y}\right)+c_{y}\\ BB_{\text{width}}=C_{w}e^{p_{x}}b_{h}=C_{h}e^{th} \end{array}\right., \end{array}$$

where (*p*_*x*_, *p*_*y*_, *p*_*w*_, *p*_*h*_) are the image center points and (*C*_*w*_, *C*_*h*_) are the bounding box center points.

The article "Early Detection of Forest Fire Using Mixed Learning Techniques and UAV" was published in 2022. Journal: Comput Intell Neurosci.

Onboard IR sensors are cast to find the heat distribution in the forest farm and then generate unichannel 2D images. The forest fire is classified into three different regions based on the temperature of the fire; it can be detected from the UAV by using highly accurate IR sensors that measure the intensity of forest fire pixels and analyze the region they fall under. The brightness of the pixels is converted into a graph, and the local maxima are considered the high-intensity region [12]. This histogram-based segmentation of pixels helps in finding the regions of fire, by taking the advantage of Otsu method. This method is defined to find a threshold that can minimize the intraclass variance as a weighted sum as follows:

(7) $$\begin{array}{c} \sigma_{w}^{2}\left(k\right)=\omega_{a}\left(k\right)\sigma_{a}^{2}\left(k\right)+\omega_{b}\left(k\right)\sigma_{b}^{2}\left(k\right), \end{array}$$

where the class probabilities are *ω*_*a*_  and *ω*_*b*_ (foreground and background) given by a threshold value and *k*, *σ*_*a*_^2^, and *σ*_*b*_^2^ are variances of both the classes.

Probabilities of classes *a* and *b* are calculated through *h* histograms are as follows:

(8) $$\begin{array}{c} \omega_{a}\left(k\right)=\sum_{j=0}^{k-1}p\left(j\right),\\ \omega_{b}\left(k\right)=\sum_{j=k}^{h-1}p\left(j\right). \end{array}$$

Intraclass variance is minimized to maximize interclass variance. The architecture of YOLOv4 tiny is shown in Figure 6.

#### 3.2.2. Prediction of the Possibility of Forest Fire

When UAV is patrolling over the forest region, it observes for the forest fire; if the fire is found, it drifts to that affected area and broadcasts all the data to the ground station and then helps the people extinguish the fire. If there is no fire in the forest, then UAV tries to find the possibilities of forest fire in that region. In general, forest fire is caused either by man-made errors or natural errors. The man-made errors that lead to forest fire are campfires that are not completely turned off, used and thrown mosquito coils, the smoked cigarettes remain, and tribal traditions related to fire. The natural causes that lead to forest fire are lightning [6, 7, 34], combustion of dry vegetation, and volcanic activities. UAV predicts the occurrence of forest fire based on any of the above-stated situations [35]. UAV finds the possibilities of fire such as oxygen, fuel, and heat (shown in Figure 7), while it is patrolling and transmits the results to the ground station.

The article "Early Detection of Forest Fire Using Mixed Learning Techniques and UAV" was published in 2022. Journal: Comput Intell Neurosci.

### 3.3. 3D Modeling of Forest Fire

3D modeling of the forest-fire-affected area helps the ground station to diagnose and analyzes the situation for extinguishing the fire and helps know the direction of the forest fire; this information is very crucial and reduces the time of extinguishing. Existing techniques for forest fire modeling are empirical and enhancement of the modeling is needed [36]. The motivation for generating a 3D forest fire model is from photogrammetric research, which enables us to generate 3D models from images with high accuracy. In this work, much effort is spent on the creation of 3D images and LiDAR.

#### 3.3.1. Construction of 3D Forest Fire Modeling

The spatial resection technique of photogrammetry is used to estimate the position of the trees in the forest by measuring evenly distributed feature points across the 2D images of the forest. The recovery of positions of tress from various directions is called “relative orientation.” Many works have been done using pixel correspondence from scaled tree positions. Recent developments have been made to generate 3D models using the 2D images using LiDAR for outdoor 3D modeling. In this work, we have adopted some of the techniques from [33]. Unlike well-designed interior images, outdoor areas such as forest, farms, and parks contain many objects. Due to relative positioning constraints for data acquisition, sampling of the surfaces is difficult using the traditional methods. Orientation of the images and distance between the tress and other objects can be easily done using LiDAR. To deal with the inconsistency of the data bottom-up approach is used. LiDAR-generated 2D images are collected perpetually from the LASER while flying in forest areas at a high speed.

#### 3.3.2. Terrestrial Image-Based 3D Modeling

Along with accurate orientations methods, tie point measure, and adjusting bundles allow sensor calibrations. Once the images are aligned, the surface measure is performed using automated procedures. Automatic photogrammetric matching algorithms are advanced and use multiple image inputs. Dense point clouds are developed using these methods and often ignore geometric constraints using smoothing. The results are shown in Figure 8.

The article "Early Detection of Forest Fire Using Mixed Learning Techniques and UAV" was published in 2022. Journal: Comput Intell Neurosci.

## 4. Experiments and Results

This model is first trained on a desktop and later loaded into UAV-CPU for testing. It is trained over 100 images for 50,000 steps each. The performance of the UAV is shown in Table 2. The comparison table of existing works and the proposed model is given in Table 3.

YOLOv4 tiny has acceptable FPS on the UAV CPU and achieves real-time detection and analysis. Few of the augmentation techniques such Mix-up and Mosaic are performed to generate the random image pairs from training data. The convolution layer in the network has good performance in detecting smaller parts of images as shown below.  Figure 9 shows that the UAV is able to detect the fire from low light intensity regions also using the Otsu method, but the high smoke zones are misclassified as the high fog zones, and fire is not detected in such cases. The model is able to detect fire in ale environmental conditions such as rainy, sunny, snow, and so on, and the training data of the model contains all three examples in equal proportion to avoid variance and bias. The other parameters such as the wind speed and temperature of the regions are analyzed, and fire is detected in such cases. Therefore, in order to improve accuracy in the high smoke zones, we used IR sensors; by utilizing the optical flow, fire is easily detected. The experimental results obtained demonstrate that the model is capable of detecting forest fires and flame regions, 3D modeling of the affected, area and forest fire tracking with satisfactory results, while the problem of using satellite imagery and low-level performance is significantly reduced as well.

The 3D models of forest fire as shown in Figures 9(a) and 9(b) are made from the predicted models. Testing results are shown in Figures 9(c)–9(f). The obtained results are worth noting and help in the analysis of the affected area.

## 5. Conclusion and Future Scope

Evolution emerges in the processing, computation, and algorithms. This strives many researchers to pay attention in many domains where they work in the processing of surveillance video streams so that abnormal or unusual actions could be detected. The usage of UAVs is recommended in the detection of forest fire due to the high mobility and ensures the coverage areas at various altitudes and locations at a low cost. Hence, an efficient and scalable UAV is used for detection. This work aims in developing the 3D model for the captured scene. YOLOv4 tiny network is deployed to detect the fire. The accuracy of the detection rate achieved through this model is 91%. The proposed model outperforms the other existing techniques in terms of detecting in the early stage. However, this model is sensitive to the forest with dense fogs and clouds. This is because smoke appears as the same as fog, and the model may misclassify the fog as smoke. As our future works, focus to meet practical detection and meet the necessity of early detection including the generation of the mixed reality model of the forest fire area that gives more information, and prevention analysis will be made easy. The 3D modeling techniques presented in this paper can also be extended to various natural disaster prediction models.

The article "Early Detection of Forest Fire Using Mixed Learning Techniques and UAV" was published in 2022. Journal: Comput Intell Neurosci.

## Figures and Tables

**Figure 1:** Proposed architecture flow.

**Figure 2:** Categorization of navigation features of UAV.

**Figure 3:** Structure of main modules.

**Figure 4:** Digital anemometer manifold with CPU, IR sensors, and 12 k camera.

**Figure 5:** (a) CBL – combination of convolutional layer, batch-normalization layer, and leaky ReLU layer and (b) CBM – combination of convolutional layer, batch-normalization layer, and mish activation function.

**Figure 6:** The architecture of YOLOv4 tiny.

**Figure 7:** The fire triangle represents the three major components (oxygen, heat, and fuel) that are necessary to generate a fire.

**Figure 8:** Generated 3D model of the forest fire.

**Figure 9:** (a) Sample 3D models of a forest fire, (b) sample 3D models of a forest fire, and (c)–(f) testing results with the developed UAV model.

**Table 1:** Specifications of the onboard equipment and masses.

S. No.	Component	Specification	Mass in grams
1.	Motor (*x*4)	T motor *u* power u5 400 kv	815
2.	Battery	6s-hv (lihv) 25,000 ma (22.8v)	1,568
3.	12 K Camera (with IR)	Blackmagic ursa mini pro 12 k	2,742
4.	Anemometer	Breezesonic 345P-4 R	300
5.	Sensors	—	600
6.	Structure	DJI	100
7.	Others (with CPU)	—	700
8.	Total payload		6,825

**Table 2:** Performance metrics of the proposed model.

S. No.	Parameter	Result
1	mAP@0.5	85.36%
2	mAP@0.75	82.45%
3	Average_IOU	83.17%
4	Precision	0.93
5	Recall	0.89
6	F1-score	0.91

**Table 3:** Performance comparison of proposed model.

S. No.	Metric	[11]	[12]	[2]	Proposed
1	Accuracy	87%	86.7%	89%	**93.3%**
2	Precision	0.87	0.86	0.89	**0.93**
3	Recall	0.78	0.81	0.83	**0.89**
4	F1-score	0.86	0.87	0.89	**0.91**

## Data Availability

The data that support the ﬁndings of this study are available from the corresponding author upon request.
